# Values of Contrast-Enhanced Ultrasound in Classification and Diagnosis of Common Bile Duct and Superficial Organ Lesions under Compression Algorithm

**DOI:** 10.1155/2021/9577440

**Published:** 2021-09-29

**Authors:** Yezhao Li, Caihong Zhao, Minpei Qin, Xia Zhang, Haizhen Liao, Haiqing Su

**Affiliations:** Department of Ultrasound, Minzu Hospital of Guangxi Zhuang Autonomous Region, Affiliated Minzu Hospital of Guangxi Medical University, Nanning 530001, China

## Abstract

This work aimed to investigate values of contrast-enhanced ultrasound (CEUS) under DEFLATE in the classification and diagnosis of the common bile duct and superficial lymphoid lesions. 88 patients with lower common bile duct lesions and 126 patients with superficial lymphoid lesions were selected as the subjects investigated and examined by CEUS under DEFLATE to compare characteristics and diagnostic efficiency of CEUS in different types of lesions. The time-intensity curve (TIC) was for quantitative analysis on CEUS results. The results showed that there were statistically significant differences in the comparison of time to peak (TTP), area under the curve (AUC), and gradient (Grad) of common bile duct walls in patients from the malignant group (*P* < 0.05), while the comparison of three indicators of patients in the benign group was not statistically remarkable (*P* > 0.05). In addition, there were statistically great differences in TTP, AUC, and Grad among patients in the benign and malignant groups (*P* < 0.05). The sensitivity, specificity, accuracy, and positive/negative predictive value of CEUS + ultrasound (US) in the diagnosis of benign and malignant lymph nodes were 92.83%, 87.14%, 89.54%, 91.23%, and 86.43%, respectively. The values of maximal intensity (*I*_max_) in the reactive hyperplasia group (group A), lymphoma group (group B), and metastatic lymph nodes group (group C) were compared, showing statistical differences (*P* < 0.05). The TTP and AUC of group B were higher than those of groups A and C, respectively (*P* < 0.05), and the base-to-peak ascending slope (*K*_UP_) and the absolute value of the semidescending slope (*K*_DOWN_) in group C increased hugely compared to group A (*P* < 0.05). It indicated that CEUS examination under DEFLATE could be applied in the qualitative diagnosis of lower common bile duct lesions and superficial lymphoid lesions, which was worthy of clinical application.

## 1. Introduction

The lesions located in the lower common bile duct usually include a variety of lesions such as stone inflammatory stenosis and tumor, which often cause biliary obstruction [1]. Compared with other imaging diagnostic methods, US examination has become the preferred method for obstruction lesions due to its convenient operation and low cost. Although the conventional US can also play an important role in the diagnosis of lower common bile duct lesions, it is easy to be affected by gastrointestinal gas; thus, it is difficult to give an accurate assessment of lower common bile duct lesions. Contrast-enhanced ultrasound (CEUS) is a new examination technology developed based on US technology, which is a major innovation of US technology [2]. With the rapid development of US contrast agents, liver, kidney, and bile duct imaging has been greatly enhanced by CEUS, and CEUS is now widely applied in abdominal and small organ diseases [3, 4]. CEUS technology can not only increase the display rate of lower common bile duct lesions but also clearly observe the enhancement speed and intensity of tissues or tumors. It is a critical tool to assist doctors in the diagnosis of lower common bile duct lesions. Therefore, the identification of lower common bile duct lesions with CEUS technology can provide more accurate and valuable information for subsequent clinical treatment and survival prognosis assessment. CEUS was first used for the diagnosis and differentiation of liver or heart diseases. Due to its continuous development and maturity, CEUS is gradually applied to the diagnosis of superficial organ lesions, such as thyroid, breast, and lymph node [5, 6]. There are differences in pathophysiological basis on different types of lymphoid lesions, the differentiation of benign and malignant lymph nodes is of great significance for the diagnosis and prognosis analysis of tumor diseases, and US examination is the preferred diagnostic method for superficial lymphoid lesions [7]. CEUS has a marked advantage in the qualitative study of benign and malignant enlarged lymph nodes in contrast to the conventional US and Doppler US imaging. The blood perfusion and microvascular distribution in lymph nodes can be observed clearly and in real time through CEUS, which provides more abundant information for doctors' subsequent diagnosis [8]. Thus, the classification and differentiation of lower common bile duct lesions and superficial lymphoid lesions by CEUS have great meanings for the clinical diagnosis of this disease and the selection of subsequent treatment options.

Data compression refers to the application of an appropriate data compression algorithm to process redundant data, so as to achieve data compression, which can not only increase the internal storage space of the device but also extend the working time to effectively improve the detection efficiency of the device [9]. Therefore, US data compression is one of the key links to promote the working efficiency of US equipment. Lossless compression means that complete original data information is retained during data compression without loss of information, and the decompression algorithm can be adopted to recover the original data, which is suitable for all kinds of scenarios requiring the retention of ultrasonic detailed data [10]. As a lossless compression algorithm, DEFLATE is an improved version of Lempel-Ziv 1977 compression format (LZ77), which is widely applied in a variety of real-time compression scenarios.

Therefore, DEFLATE was employed to compress CEUS data and analyze its compression performance and speed. Moreover, patients with lower common bile duct lesions and superficial lymphoid lesions were selected as the subjects investigated, respectively. By analyzing characteristics and diagnosis efficiency of different pathological types in CEUS, the application value of classification and diagnosis for abdominal and superficial organs were further discussed under DEFLATE of CEUS.

## 2. Materials and Methods

### 2.1. Contrast-Enhanced Ultrasound Diagnosis of Lower Common Bile Duct Lesions

A total of 88 patients with lower common bile duct lesions, admitted to the hospital from October 2018 to October 2019, were selected and grouped into a benign group (32 patients) and a malignant group (56 patients) based on the pathological results. Meanwhile, 30 healthy volunteers were selected and grouped into a control group. The criteria for inclusion were defined to include patients who had more than 5 mm maximum diameter of lesion, had received US examination, had good image quality, and were able to cooperate with doctors to complete the examination of respiration, posture, and so on. The criteria for exclusion were defined to include patients younger than 18 years or older than 80 years, suffering from pulmonary insufficiency, in pregnancy or lactation period, and allergic to the contrast agent. This experiment had been approved by the Ethics Committee of the hospital, and all the patients contained in the experiment had known about the experiment and agreed to it.

Patients drank 1,000 mL of water before the examination. Their lesion sites were scanned by conventional US and color Doppler US to observe the morphology, size, echo characteristics, and surrounding tissues of lesion sites. After that, CEUS mode was activated, and patients were instructed to breathe calmly to ensure the quality of the obtained best sections of contrast-enhanced imaging. Sulfur hexafluoride was selected as the contrast agent, and 0.9% sodium chloride (NaCl) was added into it to prepare suspension that was extracted 1.5 mL each time. When the timing of the instrument was started, an appropriate amount of contrast agent was quickly injected into the peripheral vein. Patients held their breath for 10 seconds before the arterial phase and breathed calmly for 10 seconds after the arterial phase. When the contrast agent completely subsided, the observation was stopped and the dynamic graphs within 120 seconds were stored.

TIC was used for the quantitative analysis of CEUS in and around the lesions. The region of interest (ROI) was selected and delineated based on lesion size. TIC were drawn to record various indicators by the instrument's own CEUS software. Three indicators, namely, TTP, AUC, and Grad, were selected for subsequent analysis.

### 2.2. Superficial Lymphoid Lesions Diagnosed by Contrast-Enhanced Ultrasound

126 patients with superficial lymphoid lesions, admitted to the hospital from October 2018 to October 2019, were selected to undergo US examination. There were 72 males and 54 females with an average age of 51.25 ± 15.26 years. The experiment had been approved by the Ethics Committee of the hospital, and all patients included in the study had signed informed consent. The criteria for inclusion were patients who were over 18 years old, had contraindication of CEUS, and had pathological results that were obtained by a needle biopsy or surgery. The criteria for exclusion were patients who had poor-quality CEUS images, were observed for less than 90 seconds through CEUS, had incomplete pathological results, and did not suffer from tuberculosis in TIC analysis.

All the patients had conventional US examination in advance, to mainly observe the grayscale of the target lymph nodes and color Doppler ultrasonic characteristics. After that, the patients had a CEUS examination combined with low mechanical index imaging technology. Besides, the mechanical index was set within the range of 0.03–0.07, and posterior lymph nodes were regarded as the focus of the image. Contrast agent SonoVue was selected, which had a white freeze-drier power shape, to be added with normal saline for adequate dissolution, to prepare emulsion microbubble suspension. 2.5 mL of the contrast agent was injected into the median vein of a patient, and then, 10 mL of normal saline was applied to rapidly wash pipe. A timer was started as soon as the beginning of contrast agent injection, dynamic image with the length of about 3 minutes was obtained and stored. Two experienced sonographers were selected to diagnose lymph nodes as benign or malignant based on the ultrasonic image. The patients were divided into a benign group (including group A and a tuberculous lymphadenitis group (group D)) and a malignant group (including groups B and C) based on the criteria of US-mediated puncture or surgery, to calculate their sensitivity, specificity, accuracy, and positive/negative predictive values.

SonoLiver software was applied to analyze the CEUS images, and lymph nodes were regarded as ROI to draw TIC, to obtain indexes such as RT, TTP, mean transit time (mTT), and *I*_max_. In addition, *K*_UP_ and *K*_DOWN_ were calculated, and AUC was obtained by Qontra Xt software.

### 2.3. Lossless Compression Algorithm of Ultrasonic Data

Ultrasonic data should be preprocessed before compression. According to different classification characteristics of ultrasonic data, preprocessing methods were also different. The grass wave data were preprocessed with smooth processing, and the defect wave data were preprocessed with differential processing. After the grass wave data were smoothed, the signal became smoother, the burr decreased, and the information entropy of the grass wave signal decreased accordingly, to facilitate the subsequent compression processing operation. If two peaks met the requirements and the directions of two adjacent peaks were opposite, the principle of “appear first, process first” was followed. After the first peak was smoothed, the second peak would disappear. The method of differential processing was for the defect wave. The amplitude value range of defect wave was relatively wide and the data information entropy was relatively large. After differential processing, the signal amplitude information was converted into the amplitude change information, as shown in

(1) $$\begin{array}{c} M\left(i\right)=\left\{\begin{array}{cc} A\left(i\right)-A\left(i-1\right), & i>1,\\ A\left(i\right), & i=1. \end{array}\right) \end{array}$$

In equation (1), *A* represents the original signal, *M* stands for the processed signal, and *i* expresses the signal number.

The calculation method of data information entropy is shown as follows:

(2) $$\begin{array}{c} S\left(i\right)=-\underset{i}{\sum }P\left(X_{i}\right)\log_{2}\;P\left(X_{i}\right). \end{array}$$

In equation (2), *S* stands for the information entropy and *P* and −log_2_  *P*(*X*_*i*_) express probability and self-information of *X*_*i*_, respectively.

DEFLATE was mainly composed of two coding methods (Huffman and LZ77), and the coding process is shown in Figure 1. After the raw data was entered, LZ77 encoding was first applied to generate Literal, Distance, and Length. Then, Huffman coding was employed to compress and process Distance elements to obtain DIST data rate and corresponding Huffman code table. Literal and Distance elements were combined to adopt the same operation as Distance elements to obtain LIT data rate and corresponding Huffman data table. After that, the Huffman data table was compressed, CL sequence was adopted, and SQ sequence was obtained after CL run-length coding. After its coding was compressed, the SQ data rate and the corresponding Huffman code table were obtained, and the CCL data rate was obtained after further processing.

The evaluation criteria for compression algorithms included compression ratio (CR), relative root mean squared error (R^2^MSE), algorithm complexity, and correlation coefficient *r*. CR referred to the proportion of the number of bytes after compression in the number of bytes of raw data, and the following equation could be adopted to calculate *CR*:

(3) $$\begin{array}{c} \text{CR}=\frac{N_{\text{after}}}{N_{\text{before}}}\times 100\%. \end{array}$$

*R* ^2^ *MSE* represents that the difference between compressed restored data and raw data, as shown in the following equation:

(4) $$\begin{array}{c} {\text{R}}^{2}\text{MSE}=\sqrt{\frac{\sum_{i=0}^{N}{\left(X\left(i\right)-X^{\prime }\left(i\right)\right)}^{2}}{\sum_{i=1}^{N}X^{2}\left(i\right)}}\times 100\%. \end{array}$$

In equation (4), *X* (*i*) and *X′*(*i*) stand for the raw restored data and compressed restored data, respectively.

*r* expresses the correlation between the restored data and raw data after compression, which is represented as follows:

(5) $$\begin{array}{c} r=\frac{E\left(X\left(i\right)X^{\prime }\left(i\right)\right)-E\left(X\left(N\right)X^{\prime }\left(i\right)\right)}{\sqrt{D\left(X\left(i\right)\right)}\sqrt{D\left(X^{\prime }\left(i\right)\right)}}. \end{array}$$

In equation (5), *E* (*X*) and *D* (*X*) represent mathematical expectation and variance, respectively.

*CR*, *R*^2^*MSE*, and *r* are all evaluation indexes at the mathematical level. However, the evaluation of compression algorithm complexity was indispensable in practical application, and indirect quantization representation was usually expressed by compression speed and decompression speed.

### 2.4. Statistical Analysis

SPSS20.0 software was used for statistical analysis. The measurement data were expressed as mean ± standard deviation, and *t*-test was adopted to compare the differences among the groups. Besides, the measurement data were represented as percentage, and the *χ*^2^ test was applied to compare the differences among the groups. If *P* < 0.05, the difference was statistically significant.

## 3. Results

### 3.1. Results of Data Compression Examined by Ultrasound under Compression Algorithm

The run-length encoding (RLE) [11], Huffman [12], and DEFLATE were employed to compress grass wave and defect wave data.  Figure 2 shows that CR of defect wave data obtained by different algorithms was higher than the ratio of grass wave data. The CR of grass wave data processed by RLE was markedly better than the ratio of defect wave data; CR of defect wave data processed by DEFLATE was the lowest; and CR of grass wave data processed by Huffman was the highest. Based on the above results, the compression effect of DEFLATE was better than the other two algorithms.

Under the two different platforms, the compression speed of each algorithm was lower than its decompression speed, and both the compression and decompression speed of RLE were the highest, while both the compression and decompression speed of DEFLATE were the lowest, as shown in Figure 3.

To sum up the above results, the speed of RLE, Huffman, and DEFLATE could all meet the real-time compression requirements in the personal computer (PC) platform, so DEFLATE with the best CR was selected. For the embedded platform, the compression speed of DEFLATE was too low to meet the requirements of real-time compression. Therefore, a balanced algorithm combination was selected; namely, RLE and DEFLATE were applied to compress grass wave and defect wave data, respectively.

### 3.2. The Contrast-Enhanced Ultrasound + Ultrasound Diagnosis of Lower Common Bile Duct Lesions

The results of patients' conventional US examination revealed that the lesions were located in the lower segment of the common bile duct, and lesions were 8 × 8 × 8 mm^3^–30 × 32 × 32 mm^3^ with an average size of 15.6 ± 6.4 mm and a maximum diameter of 10–32 mm. The average maximum diameter of lesions was 22.3 ± 8.5 mm in patients from the malignant group, and there were 12 patients with isoechoic or hyperechoic and 44 patients with hypoechoic. The average maximum diameter of lesions in patients from the benign group was 13.8 ± 8.3 mm with 8 patients of hyper echo and 24 patients of hypo echo.

In the benign group, the lesions of 5 patients showed high enhancement in the arterial phase, among which lesions of 4 patients expressed synchronous regression in the venous phase compared with the bile duct wall and the lesion of 1 patient had a faster clearance rate compared to the bile duct wall and showed low enhancement. There were lesions of 23 patients representing isoenhancement in the arterial phase, among which lesions of 19 patients had the clearance rate synchronized with the bile duct wall and expressed isoenhancement, and lesions of 4 patients had faster clearance rate compared with the bile duct wall in the venous phase and showed low enhancement, as shown in Figure 4(a).

In the malignant group, the lesions of 26 patients presented high enhancement in the arterial phase, among which lesions of 24 patients presented low enhancement in the venous phase and showed faster clearance in contrast to the bile duct wall, and lesions of 2 patients presented isoenhancement and had clearance synchronized with the common bile duct wall. There were lesions of 4 patients with isoenhancement in the arterial phase, lesions of 2 patients with low enhancement in the venous phase, and lesions of 2 patients with isoenhancement in the venous phase. In both phases, lesions of 3 patients showed low enhancement (Figure 4(b)).

The comparison results of CEUS indicators (TTP, AUC, and Grad) between lesions of patients in the benign group and surrounding bile duct walls are shown in Figure 5. The differences in CEUS indicators (TTP, AUC, and Grad) between lesions of patients in the benign group and surrounding bile duct walls were not marked with statistically obvious meanings (*P* > 0.05).  Figure 6 indicates the comparison results of CEUS indicators (TTP, AUC, and Grad) between lesions in the malignant group and surrounding bile duct walls. The TTP of lesions in the malignant group was remarkably lower than that of the surrounding bile duct walls (*P* < 0.05), while AUC and Grad of lesions in the malignant group were greatly higher than those of the surrounding bile duct wall (*P* < 0.05).

The comparison of CEUS indicators (TTP, AUC, and Grad) among patients in the benign and malignant group is shown in Figure 7. TTP of patients in the malignant group was sharply lower than that of the benign group (*P* < 0.05), while AUC and Grad of patients in the malignant group were dramatically higher than those of the benign group (*P* < 0.05).  Figure 8 illustrates the results of comparison of CEUS indicators (TTP, AUC, and Grad) of surrounding bile duct walls in patients from the control, benign, and malignant group. Besides, the comparison of TTP, AUC, and Grad of surrounding bile duct walls in patients from the three groups was not statistically substantial (*P* > 0.05).

### 3.3. Superficial Lymphoid Lesions Diagnosed by Contrast-Enhanced Ultrasound + Ultrasound

Pathological results demonstrated 126 patients with superficial lymphoid lesions including 52 patients in the benign group (18 patients with tuberculous lymphadenitis and 34 patients with reactive hyperplasia) and 74 patients in the malignant group (23 patients with lymphoma and 51 patients with metastatic lymph nodes).  Table 1 shows the sensitivity, specificity, accuracy, and positive/negative predictive values diagnosed by CEUS. Moreover, the CEUS images of superficial lymphoid lesions are shown in Figure 9. In the benign group, the image of a patient with reactive hyperplasia shows uniform enhancement (Figure 9(a)) from center to periphery (Figure 9(b)). Figure 9(f) indicates that the image of a patient with tuberculous lymphadenitis presents uneven circular enhancement. In the malignant group, the image of a patient with metastatic lymph nodes shows the enhancement from periphery to center (Figure 9(c)) and manifested as a nonhomogeneous enhancement (Figure 9(d)), while the image of a patient with lymphoma presents as mixed enhancement with snowstorm shape (Figure 9(e)).

Figure 10 demonstrates that the RT and mTT of patients in groups A, B, and C were not extremely different (*P* > 0.05), while there was statistical meaning in *I*_max_ of the three groups (*P* < 0.05). TTP of patients in group B was higher than that of group C (*P* < 0.05). K_UP_ and K_DOWN_ of the patients in group C increased obviously in contrast to group A (*P* < 0.05), and AUC of the patients in group C was significantly higher than the value of groups A and B (*P* < 0.05), as shown in Figure 11.

## 4. Discussion

DEFLATE was applied to CEUS image processing and the results showed that the compression effect of DEFLATE was superior to that of RLE and Huffman, which was consistent with the research results of Bras and Velden [13], indicating that CEUS based on DEFLATE could increase the internal storage space of ultrasonic equipment to improve the detection efficiency. In this study, CEUS was applied to diagnose the lesions in the lower segment of the common bile duct. It was found that there were 25 patients with isoenhancement and 7 patients with high enhancement at the arterial phase in the benign group; and there were 8 patients with isoenhancement, 46 patients with high enhancement, and 2 patients with low enhancement at the arterial phase in the malignant group. This revealed that CEUS could effectively diagnose the benign and malignant lower common bile duct lesions, which is an effective imaging method for qualitative diagnosis of the lesions. The results showed that the differences in TTP, AUC, and Grad of lesions in the malignant group and common bile duct walls were statistically obvious (*P* < 0.05), while there were no statistically considerable differences in TTP, AUC, and Grad of lesions in the benign and malignant group (*P* > 0.05). AUC reflects the blood flow and the number of blood vessels at the lesion site. The AUC of lesions in the malignant group were higher than those of the benign group and surrounding normal bile duct walls because the microvessels inside the bile duct carcinoma were rich and densely distributed, and the bile duct carcinoma was a lesion rich in blood supply and had relatively more blood flow. The blood supply in the diseased area was more abundant than that in the normal bile duct wall, and the intervascular accesses were more complex so that the peak time was relatively short. However, when Grad of the malignant group was high, the malignant tissues grew rapidly and the blood vessel wall was easy to be damaged, to easily result in an arteriovenous short circuit [14].

Liu et al. [15] found that the sensitivity, accuracy, and positive/negative predictive values of conventional US in differentiating benign and malignant lymph nodes were 64.1%, 65.2%, 47.2%, and 66.7%, respectively, while the corresponding values of CEUS were 93.6%, 75.7%, 73.7%, and 83.9%, respectively. In addition, the sensitivity, specificity, accuracy, and positive/negative predictive values of CEUS + US in the diagnosis of benign and malignant lymph nodes were 92.83%, 87.14%, 89.54%, 91.23%, and 86.43%, respectively, which were in line with the results of Liu et al. [15]. The results of the study showed that there were statistical meanings in the comparison of *I*_max_ of patients from groups A, B, and C (*P* < 0.05). The TTP of patients in group B was extremely higher than that of group C (*P* < 0.05), K_UP_ and K_DOWN_ of patients in group C were obviously higher than those of group A (*P* < 0.05), and AUC of group B increased hugely in contrast to groups A and C (*P* < 0.05). Besides, RT and PI of patients in group A were markedly higher than the values of group B (*P* < 0.05). Therefore, it indicated that CEUS could effectively classify and diagnose superficial lymphoid lesions, which was consistent with the findings of Nie et al. [16].

## 5. Conclusion

Patients with the lower common bile duct lesions and superficial lymphoid lesions were taken as subjects investigated. CEUS based on DEFLATE was applied to analyze the CEUS characteristics and diagnostic efficiency for different lesion types. The results indicated that the DEFLATE-based CEUS proposed in this study could classify and diagnose the lower common bile duct lesions and superficial lymph nodes, which had reliable clinical application value. However, there were still some shortcomings in the study. For example, the number of subjects investigated was limited and distributed unevenly; many factors were affecting the morphology and indexes of TIC; and it was necessary to determine whether TIC could be considered as a standard for differentiating benign and malignant lymph nodes by further study. In subsequent studies, the number of samples could be increased and other TIC influence indicators should be supplemented for further research and analysis. In conclusion, the results of the study provided a critical basis for the imaging diagnosis of abdominal and superficial organ lesions.

## Figures and Tables

**Figure 1:** Flowchart of DEFLATE.

**Figure 2:** Comparison of compression performance of different algorithms.

**Figure 3:** Comparison of the performance of different compression algorithms in the two different platforms. (a, b) The comparison of the performance of 3 compression algorithms in the PC and embedded platform.

**Figure 4:** CEUS images of lesions located in the lower common bile duct. (a, b) The images of benign and malignant lesions, respectively.

**Figure 5:** Comparison of CEUS indicators of lesions in the benign group and surrounding bile duct walls. (a–c) The comparisons of TTP, AUC, and Grad, respectively.

**Figure 6:** Comparison of CEUS indicators between malignant lesions and surrounding bile duct wall. (a–c) The comparisons of TTP, AUC, and Grad, respectively; ^*∗*^*P* < 0.05 in contrast to malignant lesions.

**Figure 7:** Comparison of CEUS indicators of patients in the benign and malignant group. (a–c) The comparisons of TTP, AUC, and Grad, respectively; ^*∗*^*P* < 0.05 in contrast to the malignant group.

**Figure 8:** The comparison of CEUS indicators of surrounding bile duct walls in patients from the three groups. (a–c) The comparisons of TTP, AUC, and Grad, respectively.

**Figure 9:** The CEUS images of superficial lymphoid lesions. (a, b) Images of a patient with reactive hyperplasia; (c, d) images of a patient with metastatic lymph nodes; (e) the image of a patient with lymphoma; (f) the image of a patient with tuberculous lymphadenitis.

**Figure 10:** Comparison of CEUS indexes (a) RT, (b) TTP, (c) mTT, and (d) Imax of the patients in group A, B, and C. ^*∗*^ and # stand for *P* < 0.05 in contrast to groups B and C, respectively.

**Figure 11:** Comparison of K_UP_, K_DOWN_, and AUC of the patients in the three groups (^*∗*^ and # stand for *P* < 0.05 in contrast to groups A and C) respectively).

**Table 1:** Diagnosis results of CEUS + US.

	Sensitivity (%)	Specificity (%)	Accuracy (%)	Positive predictive value (%)	Negative predictive value (%)
CEUS + US	92.83	87.14	89.54	91.23	86.43

## Data Availability

The data used to support the findings of this study are available from the corresponding author upon request.
